# Exploration of Happy Learning for College Students with the Integration of Thinking Visualization and Action Learning in the Internet + Environment

**DOI:** 10.1155/2022/9039630

**Published:** 2022-09-01

**Authors:** Zhen Han

**Affiliations:** Mental Health Education Center, North China University of Water Resources and Electric Power, Zhengzhou 450045, Henan, China

## Abstract

Under the background of networked education, the subjective behavior in the field of education, the interaction between teachers and students, and the educational environment in which the subject is located have all had a comprehensive impact on the teaching mode of mental health courses in colleges and universities. In recent years, the teaching research and practice related to “action learning” and “thinking visualization” have been deepening, and more papers, monographs, and training activities related to them have been deepened. Thinking is a complex cognitive process, and students' positive and critical thinking attitude plays a crucial role in improving the quality of nursing work in the future. The importance of study, our way of self-cultivation, and the foundation of our destiny is beyond words. This study explores the application and significance of college students' happy learning combined with the visualization of thinking and action learning under the background of “Internet +” from four aspects: curriculum connotation, system construction, effect analysis, and curriculum thinking, so that students can play their subjectivity in education courses and improve. The initiative and interaction of students in the classroom encourages students to not only know, feel, and experience in education courses but also dare to speak, ask, and question and be the leaders of the classroom.

## 1. Introduction

Among the many factors that affect learning, it can be seen from the main factors affecting learning in Figure 1 that learning approaches have the greatest impact on learning quality. It is a general term for the values and corresponding behaviors held by learners to complete learning tasks and achieve learning goals. Whether the learning method is appropriate directly affects the quality of students' learning and the innovation ability of one generation, several generations, and a nation [1].

The learning style determines the learning quality, which in turn affects the well-being of college students. Therefore, the school is essentially to teach students mental health knowledge through the university system, help them establish the main channel and main position of perfect and good personality, train students' mind and creativity, and guide students to develop good interpersonal relations by investigating the mental health problems of different age groups, as shown in Figure 2. To further explore a more efficient teaching mode is the main task of happy learning for college students [2]. As for the research on curriculum teaching methods, some scholars advocate building a happy learning classroom education for college students through activity-based teaching methods, cooperative classroom methods, workshop teaching models, etc., while others advocate using mental tests, character dressing, group discussion, and scene simulation. Other methods can also be used to achieve the classroom education of happy learning for college students. Some scholars have proposed introducing new classroom methods, such as flipped classroom, MOOC and other mixed classroom, and applying them to the happy classroom education for college students. According to the “three entry” demand for happy learning of college students, namely “brain, heart, and behavior,” we can focus our research perspective on the means innovation and system improvement of College students' mental health curriculum methods. According to the existing theoretical and empirical research results, in the context of “Internet +,” the research method of organically combining the scientific calculation visualization of thinking with the way of action is the most effective method to improve the classroom results of happy learning of college students [3]. Due to the influence of psychological problems, college students are prone to emotion and inattention during the learning stage, which has an important impact on college students' happy learning. In view of this, in order to better improve the ability of college students to learn happily, we plan to introduce the action learning method to strengthen the three links of early search, mid-term communication, and post-assessment in the form of team study groups, so as to improve the enthusiasm and autonomy of college students to learn happily and scientific validity.

## 2. The Connotation of College Students' Happy Learning with the Integration of Thinking Visualization and Action Learning

One of the connotations of happy learning is interest. When the interest in learning is turned into an active learning action and the pursuit of the desire for success, it will not only deepen the interest but also generate a continuous motivation for happy learning from the perception of the learning process.

The second connotation of happy learning is success, and success will bring motivation to people and become an important part of a happy life, however, failure is not exactly equal to pain. Edison's experiment to invent the light bulb was done 999 times without success, and “I found 999 times that there is no way to make a light bulb”, was his answer to 999 failures.

The third connotation of happy learning is to reduce the burden. The increasingly competitive environment and the ensuing variety of test takers have brought different degrees of pressure to learners at different stages and at different levels, and the appearance of pressure is that learners have a psychological burden [4].

### 2.1. Thinking Visualization Teaching Strategy

In practice, the teaching strategy of thinking visualization can be summarized as three basic operation steps: discovering structure, presenting structure, and transferring structure. It is based on structured thinking. Of course, many people think that there are many types of thinking, such as image thinking, epiphany thinking, inspirational thinking, and innovative thinking. Hence, they are opposed to focusing on the cultivation of structured thinking ability for students' thinking development. In fact, the emergence of this concept is caused by insufficient understanding of the nature of thinking—no matter what kind of thinking, its core is based on structure, however, the structure types are different. Some are hierarchical structures, some are linear structures, and some are mixed structure, including innovative thinking. Its essence is not random association but the optimization and reorganization of the structure. If the structure is lost, people's thinking will fall into a kind of morbid state—thinking runaway [5].

In addition, in the practice of course teaching, because each course has different scene environment and teaching characteristics during teaching, the application of the thinking map visualization teaching strategy should also fully consider the teaching characteristics of each course: in the science course represented by mathematics, emphasis should be placed on the use of “theme fishbone diagram” and “mathematical logic deduction diagram” to cultivate the learners' ability of “long-chain reasoning” [6]. In the liberal arts teaching represented by Chinese, the focus is on using “subject mind map” and “problem-solving strategy modeling” to help students improve the ability of “multilevel accurate generalization.” In addition, it is also necessary to pay attention to the unique thinking nature and development laws of different disciplines and integrate them with the thinking visualization teaching strategy. Refer to Figure 3 for the specific thinking visualization map model.

### 2.2. The Connotation of Action Learning

Action learning research is the product of the confluence of action learning and action research at the end of the twentieth century, which refers to the specialized existence of human life and its optimization activities [7]. The theory of “action learning” believes that learning activities are a series of continuous processes of action and reflection, which is the combination of structural knowledge and the four elements of questioning, reflection, and execution, emphasizing the construction of learning through the reciprocating cycle of knowledge, reflection, and action. The introduction of action learning research in the reform of college students' learning style will definitely have a profound impact on the construction of the “organism” professional development concept, the shaping of the “autonomous reform” professional development method, and the formation of a networked professional development ecology [8]. The general process of action learning can be divided into seven steps, which are specifically represented by Figure 4.

#### 2.2.1. Action Learning Research Is Conducive to the Construction of the Concept of “Organism” Professional Development

Marx's theory of “social organism” provides important theoretical support for the construction of a harmonious society and has an important guiding significance for the construction of a harmonious socialist society. “Organism” regards the world as an organism, and it focuses on the “dynamic” natural operation of the organism. The life process of the organism continuously provides feedback for the survival of the organism, and the external environment provides support for the feedback inside the organism [9]. Corrective action learning research advocates that the professional development of people in industrial and postindustrial societies should not be a one-sided development of a certain aspect (such as cognition, skill, and morality) but should be the organic advancement of spirituality, ethics, values, worldview, and practical behavior.

#### 2.2.2. Action Learning Research Is Conducive to the Formation of a Networked Professional Development Ecology

The networked professional development ecology is a professional development state in which all participants can achieve a win-win situation through collaboration [10]. Action learning research abandons the linear transfer of expertise and skills from experts to novices, while avoiding the neglect of the agency of professional development objects. It treats all those involved in action as people with professional development needs, and at the same time, it makes them equal actors, uses a combination of qualitative and quantitative research methods, learns and researches through action, experience, and reflection, implements self-management, seeks to establish a networked team with the same interests and values to achieve the unity of action and thinking, and integrates theory and practice. In this way, in a specific professional development activity, individuals can put their knowledge, skills, time, and energy into action learning and action research and process the management of interest, collaborate with others, motivate each other, and complete collaborative tasks to improve the quality of the overall work.

### 2.3. The Connotation of College Students' Mental Health Course

As a special group, college students often face various psychological pressures in daily life and study, and all kinds of psychological pressures are accumulated together, and over time, they will cause psychological obstacles. As a tianzi child, mental health is the foundation of academic achievement, career success, and happiness in life. Under the background of network teaching, behavior teaching is helpful to train learners' integration and coordination ability, and promote students' lifelong ability. It can be seen that the positive effect of behavior teaching is not only manifested in the learners' academic ability in class, but also in the cultivation and shaping of the learners' overall ability and knowledge level. Moreover, behavior teaching can also improve learners' initiative and interaction in the curriculum [11].

Thinking visualization refers to the process of presenting invisible thinking paths, structures, methods, and strategies in the form of diagrams or a combination of diagrams to make them clearly visible [12]. In layman's terms, it is to “draw” the thinking in the brain. Action learning originated from the “action learning theory” proposed by Professor Reg Revans and others in the United Kingdom. It refers to the learning and reflection process under the mutual support of group members, emphasizing the use of team spirit, teamwork, and mutual support. Support and share experiences to solve difficult problems.

It can be seen that the mental health course model for college students that integrates thinking visualization and action learning under “Internet +” means that teachers guide students to learn to actively internalize the knowledge system with the mutual support of group members, and integrate online micro-lectures with The paths, structures, methods, and problem-solving strategies of the thinking and feeling of the offline classroom are presented in the form of diagrams or a combination of diagrams to make them clearly visible, thereby effectively improving students' learning efficiency and sense of gain and improving students themselves. Knowledge system.

## 3. Exploration of College Students' Happy Learning with the Integration of Thinking Visualization and Action Learning under “Internet +”

In the “Internet +” era, we will introduce thinking visualization. In view of the learning and teaching reform in the “Internet +” era, we will face several new topics that must be considered and discussed in the college students' mental health class that combines thinking visualization and behavior learning. First of all, teachers must cultivate the ability of subject thinking and behavior learning data visualization. After having a deep understanding and skilled application, they can better guide students to practice in the classroom; secondly, the classroom scale should be limited within the most appropriate scale, and the classroom layout should be flexible and diverse (such as movable desks and chairs) to avoid students' interference with classroom teaching; finally, the content of online microcourses and offline classes should strive to improve, reasonably connect and echo, so that learners can more clearly visualize their ideas through action learning, and truly form their own classroom leaders [13]. The subjective feelings of college students' happy learning and the extent to which these feelings are helpful to college students' happy learning are shown in Table 1.

### 3.1. Teaching Objectives

The mental health course for college students, which combines the visualization of thinking and action learning under “Internet +,” aims to improve the mental health of college students and develop a healthy personality, and it is guided by the actual needs of students and the improvement of psychological literacy. At the same time, it helps improve their psychological self-help and helping skills and internalizes their mental health knowledge and skills system. At the knowledge level, this research popularizes the basic concepts of mental health to college students, guides college students to internalize mental health knowledge, and improves their own mental health knowledge system through the investigation of college students' learning motivation. Learning attitude data are shown in Figure 5. From the data in the figure, it can be seen that different learning goals have different changes in the learning status and mental health of college students, and to further study the exploration of college students' happy learning, it is necessary to deepen the research.

In the aspect of psychological teaching, the combination of cognitive visualization and action cognition can not only cultivate students' self-help ability and development ability, thus improving students' cognitive efficiency and acquisition, but also help students better understand and accept themselves, thus forming healthy and positive psychological quality and promoting students' self-improvement and development [14].

### 3.2. Course Audience

Therefore, psychological courses should not only adapt to the age characteristics and psychological development laws of contemporary college students, but also keep pace with the times, fully mobilize their enthusiasm and attention in learning, and carry out online and offline in the context of “Internet +.” Through the multipronged curriculum, the coverage of psychological knowledge has been greatly increased, and the shackles of time and curriculum have been broken [15]. Secondly, some traditional college students' mental health education courses only teach theoretical knowledge and ignore the guidance of students' self-cognition and perception. Some college students' mental health education courses pay attention to the combination of online and offline and focus on students. However, they ignore the guidance and practical application of students' skills and the effective integration of knowledge and skills, so that college students cannot apply what they have learned. Therefore, it is necessary to guide students to adopt the combination of thinking visualization and action learning in the course, give full play to the main role of college students, arouse their interest in learning, stimulate their active learning, and form a self-knowledge system. Students can effectively integrate knowledge and skills, enhance and improve their sense of self-acquisition, improve their psychological literacy, and promote their self-growth.

### 3.3. Teaching Design and Effects

#### 3.3.1. Teaching Content

The teaching content is adjusted. The mental health course for college students is intended to enable us determine the moral standards and practical significance of physical and mental health under the concept of “great health.” Through understanding and applying modern psychological science knowledge, we can cultivate our good social and psychological quality, international cooperation consciousness and broader vision, so as to comprehensively improve our overall psychological quality and lay a good and healthy psychological foundation for our lifelong development. Through the combination of theoretical research and psychological teaching research, it is found that some college students have corresponding problems in the fields of social adaptation, interpersonal relationship, emotion, love, learning, job hunting, and self-awareness. The classification is shown in Table 2. In order to ensure that the course content meets the actual situation of learners, this study has formed a teaching content system in seven major directions: adaptive psychology, interpersonal communication, emotional psychology, love psychology, learning psychology, job seeking social psychology, and self-development. Its home: “Freshmen's adaptation problems,” “winning friends like clouds: benign interpersonal communication,” “emotion management: I am the master of my emotional intelligence,” “love growth: love people with similar aspirations,” “adjust mentality and cope with pressure,” “understand occupation and face occupation directly” “three reflections on my body: standards and concepts of physical and mental health,” “mechanics practice: Aerobic Teaching,” “understand yourself and accept yourself,” and so on [16].

#### 3.3.2. Teaching Methods

Teaching methods. The psychological health class of college students further enhances the learners' sense of experience and acquisition through the teaching mode of organic combination of online and offline teaching, organic combination of theoretical knowledge and experience courses, and organic combination of education and training [17]. At the same time, the “Internet +” psychological classroom for college students, which integrates thinking visualization and behavior learning, not only takes the learners as the main body of the classroom, but also takes the direct feelings of the learners as the teaching basis, and uses thinking visualization and behavior to guide students. Through the combination of active exploration and active experience, the methods of classified discussion, participatory interaction, and case analysis, as well as psychological skill experience through self projection test, imagination, and relaxation, are adopted to let learners understand the physical and mental adjustment knowledge under different teaching modules, so as to effectively integrate theoretical knowledge and ability, cultivate, and improve students' practical application ability, and self-help and service to others. Finally, with the mutual support of the organization team, the students can internalize the curriculum system independently and combine the teaching ideas and content ideas, organization, thinking mode, problems, and methods of online microclass and offline class with tables or graphics. It can effectively improve students' learning effect and sense of mastery, and improve learners' own cognitive system.

#### 3.3.3. Curriculum Effect

This study used a combination of open-ended and closed-ended questionnaires to conduct surveys. 260 questionnaires were distributed in the classroom, and 247 valid questionnaires were recovered. The analysis of the results shows that 94.3% of the students are very satisfied with the mental health course model for college students that combines thinking visualization and action learning under the background of “Internet +.” Among them, 87.6% of the students believed that this course model not only consolidated some theoretical knowledge of their own psychology but also promoted their own mental health development. 93% of the students said that they would combine the psychological knowledge learned and experienced in the course with the Apply skills to study and life. 87% of students reported feeling learning to work better together and to be more proactive in facing and solving problems. 97.1% of the students indicated that this model made them feel a sense of gain and gain, and they felt that they were the main body of the class and were more willing to speak, ask questions, and share in class.

## 4. Strategies and Suggestions for College Students to Study Happily

In the context of “Internet +,” this research is the first to apply thinking visualization and action learning to college students' mental health courses. Through the thinking visualization technology, students' initiative and subjectivity in mental health courses are improved. The action learning of reflective learning and collaborative learning can enhance students' authentic experience, interaction, and subjectivity. In view of this situation, we propose some strategies on how to make contemporary college students become happy and deal with study and life efficiently, as shown in Table 3. Regarding the research on college students' mental health curriculum, it mainly focuses on the background of “Internet +” education, introduces a new concept into college students' mental health education curriculum, and innovates the teaching mode of college students' mental health education course from the technical level.

### 4.1. Keep Yourself and Make Good Use of Your Talents

The inability to maintain one's self is one of the main reasons why contemporary college students are often confused. When people see others getting good grades, they think that they cannot get high grades no matter how hard they try. Hence, they feel very inferior. They lose enthusiasm for study and life and became very decadent because of this. They spend time playing games every day and finally achieve nothing. This lesson teaches us to be ourselves at all times. William James once said, “Compared to what we should have achieved, we are actually half awake, and we use only a small part of our physical and mental resources. Constrained, we have all kinds of resources but often do not use them properly.”

### 4.2. Develop Good Study and Living Habits

The main reason for the poor efficiency of contemporary college students is that they do not develop good habits. We all know that colleges and universities have fewer courses than high schools, and the daily class time is uncertain. It makes many contemporary college students develop many bad living habits. If there is no class tomorrow morning, the students will play with their mobile phones until late. Naturally, they wake up so late in the morning that they do not even have time to eat breakfast. Hence, the person looks sluggish, confused, and has no interest in doing anything [18]. If we do not even have the passion to study and live, can we still study efficiently? Carnegie said that people will not die because of overwork, however, they will go away with debauchery and sorrow [19].” In response to this phenomenon, we should create a good environmental atmosphere. The phrase “near Zhu is red, near ink is black” illustrates the important impact of the environment on people. These environmental cues send messages to students in a very natural way. As contemporary college students, we should be full of vigor, and we should all have our own dreams like a river, which is to run to the sea. Contemporary college students should not live a busy life every day. Developing good living and study habits makes one not only healthier but also feel full and happy. Therefore, the second rule to make oneself happy and improve learning efficiency is to develop good study and living habits.

### 4.3. Do Not Get Bored with Things

When we walk into a certain class in colleges and universities, we may find that the mental state of the students is very bad. Some students are lying on the table and their movements are very lazy. Some classmates are simply playing with their mobile phones secretly. The vigor of the past seems to have disappeared. Is it because they usually have heavy academic and family work, which makes them very tired? no. The real cause of this phenomenon is fatigue. The real reason why you are bored with something is that you are not interested in it at all, or even resist it. Therefore, the main reason for the decrease of the effect of college students in class is that the learners themselves are tired of the class, or their enthusiasm for class is too low. The famous Japanese radio news analyst Katsuya Fujimoto, every morning before leaving, he said to himself in the mirror: “Fujimoto, if you want to eat something, you should do this job well. But since you have to do it, why not do it and be happy? What? Why don't you pretend to be a performer when you see your performance after you ring the doorbell? In short, what you do is as interesting as performing on the stage. Why don't you have some interest and enthusiasm for it?” [20]? Contemporary college students should learn to go with the flow, since everything around them cannot be changed, however, if one can insist on what one cannot change, one will eventually change oneself. Hence, one must make oneself happy and improve learning efficiency. The third rule is to not get bored with life and make learning fun.

## 5. Conclusion

In today's rapid development, contemporary college students should not follow the crowd and maintain their own style at all times. Teachers, students, and disciplines are the three elements that constitute teaching activities, and there have been many controversies surrounding the relationship between these three elements in the past teaching reform practice. Take advantage of yourself. Build your own garden, develop good study habits, and be passionate about study life. Continue to let knowledge fill the hearts and let sweat fill every day. At the same time, contemporary college students have to relax themselves in a stressful environment. In this way, we not only have a healthy body but also a happy mind. Therefore, under the background of “Internet +,” by establishing a combination of thinking visualization and action learning for college students' happy learning and exploration, students can play their subjectivity in learning and education courses, improve students' initiative and interaction in the classroom, and promote students. In the education curriculum, one must gain not only true knowledge, true feeling, and true experience but also must dare to speak, ask, and question and be the leader of the classroom. At the same time, the research on the construction of college students' happy learning course combining thinking visualization and action learning under the background of “Internet +” also has practical guiding significance for the work of college teachers.

## Figures and Tables

**Figure 1:** Main factors affecting learning.

**Figure 2:** The changing trend of mental health level of different age groups.

**Figure 3:** A map of thinking visualization attempts in learning.

**Figure 4:** The seven key steps of action learning.

**Figure 5:** The survey map of college students' learning goals and motivation.

**Table 1:** The subjective feelings of college students' happy learning.

Research project	Great help (%)	Help (%)	Some help (%)	Add 3 terms (%)
Enriched mental health knowledge	34.5	49.3	13.90	97.70
Understand the importance of mental health	34.10	47.4	15.9	97.4
Improve frustration tolerance	24.00	40.60	29.00	93.60
Learn emotion regulation	24.10	44.90	26.40	95.40
Improve cognition	27.70	43.90	23.70	95.30
Enhance interpersonal communication	21.74	38.10	32.13	91.97
Improve learning efficiency	22.20	32.10	36.00	90.30
Know yourself and others correctly	29.60	42.40	23.40	95.40
Improve personality	24.40	36.80	29.50	90.70
Treat love correctly and understand sexual knowledge	28.53	38.10	24.24	90.87
Learn how to self-regulate mental health	31.16	41.00	22.58	94.74
A more positive attitude towards life	34.90	37.70	23.10	95.70
Psychologically more adaptable to social changes	29.80	41.00	23.30	94.10

**Table 2:** University Psychological confusion classification.

Classification	The nature of mental activity	The nature of psychological conflict (xu Youxin's qualitative distinction)	Question duration (guide to principle)	Does the content generalize (main principle)	Severity of the problem (reference principle)
General psychological problems	Normal unhealthy state	Regular conflict	Within a month	Not yet generalized	Basically no impact on social function
Serious psychological problems	Normal unhealthy state	Regular conflict	Longer within three months	Generalized (similar, related stimuli can also elicit symptomatic responses)	Has resulted in mild impairment of social functioning
Neurotic psychosis (suspected neurosis)	Normal unhealthy state	Begin to deform	Longer within six months	Severe generalization (unrelated, dissimilar stimuli begin to elicit symptomatic responses)	Moderate impairment of social functioning
Neurosis	Abnormal nonpsychotic disorder	Metamorphosis conflict	Very long more than three months	Full generalization (unrelated, dissimilar stimuli continue to elicit symptomatic responses)	Severe impairment of social functioning

**Table 3:** Strategies and suggestions for college students to study happily.

Strategy	Advice
Stay away from mobile phones	Many people believe that mobile phones have become the most depleting and distracting things today. Especially in recent years, the short video platform has developed rapidly, and short videos have also made many people want to stop. Moreover, the mobile phone keeps popping up message reminders, which will always interrupt one's thinking and work. Hence, if one wants to improve one's efficiency, the first thing one should do is to stay away from the mobile phone, put the mobile phone elsewhere, and try not to take the initiative to take it during the learning process.

Choosing an environment	Many people want to watch TV shows, play games, or just lie back in bed to play with their mobile phones as soon as they enter the dormitory. Most of the day has passed. If one want to get rid of one's “procrastination”, change the learning environment. For example, if one wants to improve learning efficiency, one can go to the study room or the library. 2. Change the environment. There is no bed to interfere with one, and the surrounding learning atmosphere can better allow one to study with the peace of mind.

Make a plan	Make a plan not only to simply plan the things that need to be done on the day but also to simply arrange the time range for doing each thing and strictly follow the plan. It requires the students to have a better understanding. 3. Make a plan to promote high self-awareness and self-discipline, one must be strict with oneself in the process of completion

Appropriate pressure	Increase pressure on the self appropriately by compressing the time one has to complete a certain thing. The lesser the time one gives oneself for the task, the sooner one will complete it. For example, in the final review, many students do not start reviewing until a week or even three days before the exam. It will definitely be completed within a few days. Hence, compressing time is like getting close to the deadline for things, and one will take the initiative to do things.

Supervision of each other	In college students, procrastination is not just isolation, it is a problem faced by many students. Hence, several roommates can supervise each other. For example, when completing the task assigned by the teacher, they can start together. Multimotivation to support oneself and mutual supervision can also effectively achieve one's goals.

## Data Availability

The labeled dataset used to support the findings of this study is available from the corresponding author upon request.
